# Research on Higher English Internationalization Education Model and Evaluation Index System Based on Multi-Source Information Fusion

**DOI:** 10.1155/2021/1599007

**Published:** 2021-12-22

**Authors:** Bei Yang, Huijun Tang, Lei Mou

**Affiliations:** ^1^School of Foreign Languages and Cultures, Chengdu University, Chengdu 610106, China; ^2^School of Foreign Languages, China University of Geosciences, Wuhan 430074, China; ^3^The Office of International Cooperation and Exchange, Chengdu University, Chengdu 610106, China

## Abstract

With the continuous development of the global economy, the degree of internationalization and openness has gradually deepened. Higher English internationalization education also needs to keep pace with the times and keep pace with international development. At this time, it is necessary to build a multi-source information fusion algorithmic higher English international education model and evaluation index system to better adapt to the trend of higher English international education in the future. In the current higher English teaching process, it is necessary to change the traditional teaching concepts, change the previous teaching ideas, continuously expand the horizons, build an international and diversified English teaching training program, and actively absorb excellent education concepts from foreign excellent teaching models, which has better promoted the development of English teaching.

## 1. Introduction

English classroom education is mainly centered on the exchange activities between teachers and students. It is a system with significant social characteristics. The corresponding evaluation index system and teaching model together constitute the education level weighed by the higher English evaluation index [1–3], according to the principle of combining pre-teaching appointments and post-teaching satisfaction. At present, cloud computing, computer technology, big data analysis, and hypermedia technology are the basis for promoting the continuous development of modern information technology; it can provide English learners with virtualized teaching services and fast teaching services, which are generally interconnected, intelligent, and huge. Data-scale data information mining, image-friendly learning interface, and other data information technology services can not only effectively improve the environment of higher English teaching, but also change the previous views and learning styles of English teaching. The relationship between teachers and students can apply higher English learning to the actual era of information development, and it has become the main factor that can realize the “structural reform” of higher English education. Education itself is to cultivate high-quality people, who are useful to society. Traditional education is centered on teachers. Teachers dominate and students passively participate. Students trained in this model rarely have innovative thinking. They are obedient and dependent. Learning is not so enthusiastic, and there is rarely a rich imagination, and scientific research and creation all need imagination as a support. Therefore, cultivating students' imagination and innovating their thinking ability is the motivation and purpose of our research. Through research, it is found that multimedia education is based on traditional education, which is obviously more advantageous and can stimulate students' enthusiasm. It is full of enthusiasm for learning and let students take the lead in learning. Therefore, multimedia support education is not only a tool to assist education, but also a transformation of modern education for the improvement and reconstruction of learning methods, which is a leap in the quality of traditional education.

By constructing a higher English international education model and evaluation index system, this paper analyzes the key factors of the higher English international education system in the current information age in detail. It mainly initializes teaching information from the perspective of English teaching evaluation and analyzes the international English education in colleges and universities' level and quality.

## 2. Classroom Evaluation Health: A New Vision of “Effective Teaching” Evaluation Research

Learning is based on a certain English environment, with the help of others and multimedia, that is to say, the process of meaning construction achieved through cooperation activities between people. Therefore, in this mode, “condition, cooperation, dialogue, and meaning construction” are the four elements in the learning environment. The characteristics and functions of multimedia technology are conducive to fully embodying the four elements. In order to provide a supportive education model, it provides the necessary conditions for effective use in English classrooms. Based on the above viewpoints, the multimedia support English education model is the specific application of constructivist learning theory in multimedia English education. Multimedia support education is to teach knowledge before class in traditional classrooms, and the internalization of knowledge is to carry out work activities after the original class and then transfer to learning activities in the classroom. Combined with the concept of multimedia-supported education, a multimedia-supported education model with four stages of education preparation, memory, application analysis, and comprehensive evaluation of education was designed. Take university English as an example, try the composition, and establish higher vocational education. The college English multimedia-supported teaching model divides the college English multimedia-supported teaching into two stages: pre-education and classroom. Discussions on knowledge extraction, online learning, and classroom problem-solving are given in Figure 1. See the figure for the four links of evaluation and feedback.

The development of students is divided into two stages. The first stage is the individual differences of students. The results are different. The second stage of development is under the guidance of teachers, and students can dig out the potential level of development. Use this to verify. In the case of underachievers, some students have average grades at the beginning of their studies. As long as their teacher provides reasonable guidance, this student can make great progress. Therefore, the educational model has an important influence on the development of students. Therefore, teachers should formulate educational plans around students' learning conditions.

In the knowledge extraction link, the teacher selects the main points of knowledge according to the students' knowledge level, learning foundation, learning ability, and learning habits; determines the teaching goals, teaching difficulties, and learning tasks of each unit; and refines enlightening and guiding questions. The online learning link is under the guidance of the teacher's questions; students can watch teaching videos in groups or independently by themselves to learn the main language, sentence structure, cultural background, and text structure. At the same time, with the help of the group leader, they can understand the main knowledge points as much as possible and bring the unsolvable knowledge content to the classroom. In the classroom discussion problem link, students expand their self-learning language and culture knowledge in groups or individually and apply them to various activities and tasks of classroom teaching to promote the students to absorb, internalize, and apply the knowledge they have learned. In this link, students need to complete the exercises and exercises related to online learning tasks, as well as activities such as after-reading feelings, situational dialogues, role-playing, keynote speeches, and hot topic discussions. In addition, for common problems, teachers should organize students to collaboratively solve and summarize. For personality problems, teachers should inspire and guide students to solve them independently and give individual guidance; the evaluation feedback link is given after the completion of the first three links; then the teacher will conduct a summary evaluation of the strengths and weaknesses of the learning situation and performance and propose improvement measures and future directions for efforts. Through the implementation of this link, students can further consolidate and improve the knowledge they have learned and have a better understanding of the problem.

To accurately evaluate the internationalization of higher English education, we first need to build an evaluation model of English education model. Combining nonlinear information fusion methods and time series analysis methods, statistical analysis of the teaching ability of English international education is performed. Higher English internationalization education model and evaluation ability constraint index parameters are a set of nonlinear time series. Constructing a high-dimensional feature distribution space represents the distribution model of higher English analysis and evaluation parameters, and its main index parameters restrict the teaching ability of English international education, teachers' level, investment in educational facilities, and policy relevance. Construct differential equations and construct an information flow model that expresses the constraint parameters of English international education ranking ability [4–7].

(1) $$\begin{array}{c} x_{n}=x\left(t_{0}+n\Delta t\right)=h\left[z\left(t_{0}+n\Delta t\right)\right]+\omega_{n}. \end{array}$$

In the formula, *h* (·) is the multiple value function of the analysis and evaluation of English international education. *ω*_*n*_ is an evaluation error measurement function. In the high-dimensional feature distribution space, the solution vector of the analysis and evaluation in the English international education teaching is calculated by the correlation fusion method, and the feature training subset *S*_*i*_(*i*=1,2,…, *L*) of the education analysis and evaluation is obtained, and the following conditions are met:

1. $\Sigma =\text{diag}\left(\delta_{1},\delta_{2},\ldots ,\delta_{r}\right),\;\delta_{i}=\sqrt{\lambda_{i}},\forall i\neq j$
2. ∪_*i*=1_^*L*^*S*_*i*_=*V* − *v*_*s*_

where *x*_*n*+1_=*μx*_*n*_(1 − *x*_*n*_) indicates that the evaluation index of higher English internationalization education adopts the conjugate solution of the statistical information model, which can reach the decomposition condition *U*={*u*(*t*)*|u*(*t*) ∈ *X*, ‖*u*‖ ≤ *d*, *t* ∈ *I*} of the initial value, among which (*I*_*i*_)_*i*∈*N*_={*x*_1_, *x*_2_,…, *x*_*m*_}. For multiple variable groups, the characteristic distribution sequence *x*(*n*) corresponding to the evaluation statistics of higher English internationalization education can be used to construct a higher English internationalization education model based on the measured value of the previous teaching level.

(2) $$\begin{array}{c} c_{1x}\left(\tau \right)=E\left\{x\left(n\right)\right\}=0,\\ c_{2x}\left(\tau \right)=E\left\{x\left(n\right)x\left(n+\tau \right)\right\}=r\left(\tau \right),\\ c_{kx}\left(\tau_{1},\tau_{2},\ldots ,\tau_{k-1}\right)\equiv 0,\;k\geq 3. \end{array}$$

When *Q* = 2, the teacher's strength level and the distribution level of educational resources in the higher English classroom evaluation meet the (2 + 1) dimensional continuous letter writing condition [8–10]. In other words, the courses of English internationalization education should be analyzed and evaluated.

(3) $$\begin{array}{c} \psi_{x}\left(\omega \right)=\ln\;\Phi_{x}\left(\omega \right)=-\frac{1}{2}\omega^{2}\sigma^{2}. \end{array}$$

The exclusive analysis and evaluation data information flow model of English international education it provides an accurate data input basis for the teaching analysis and evaluation of English international education and constructs a set of scalar sampling sequence components.

The multi-source information fusion algorithm is used to analyze the big data information model of the higher English international education model and the evaluation index system, and the control objective function for constructing the prediction and estimation of the ability of the higher English international education model is

(4) $$\begin{array}{c} \underset{x_{a,b,d,p}}{\max}\sum_{a\in A}\sum_{b\in B}\sum_{d\in D}\sum_{p\in P}x_{a,b,d,p}V_{p}, \end{array}$$

(5) $$\begin{array}{c} \text{s}.\text{t}.\;\sum_{a\in A}\sum_{d\in D}\sum_{p\in P}x_{a,b,d,p}R_{p}^{bw}\leq K_{b}^{bw}\left(S\right),\;b\in B. \end{array}$$

Therefore, a specific analysis is made on the health evaluation index system of high school English teachers in the information learning environment.

## 3. The Health Evaluation Index and Measurement Analysis of College English Classroom Evaluation under the Information Environment

### 3.1. The Evaluation Index of College English Classroom Teaching System in the Information Learning Environment

According to the knowledge theory of health review, the motivation of the teaching system comes from the passage of English teachers and students in the system. The motivation of the English teaching and activity input system is mainly to promote the change of higher English international education mode, which needs to be measured indirectly through the obvious teaching mode of the outside world [11–13]. According to the analysis of the teaching process between the higher English teaching teachers and students, the types and characteristics of teaching activities are used to evaluate the health index system of higher English teachers. The higher English internationalization education model mainly prepares English teachers and English classroom education and provides special tutoring. The types of student education activities include students studying with teachers, and mutual help among students within teachers. The characteristics of higher English international teaching activities can use teacher enthusiasm and teaching. The time used by the process is measured. The characteristics of the student's learning model can be explained by the student's enthusiasm for learning and the amount of time spent on learning. The teaching enthusiasm of higher English teachers is used to evaluate the degree of effort of teachers in English teaching activities, and it is also an active psychological activity that appears in higher English teaching as a teaching model. Under the modern information, the motivation to input the evaluation system of higher teachers, in addition to the two main teaching models of teachers and students, is the evaluation basis of the evaluation system under data informatization. In the past, higher English education needed a teaching model shared by teachers and students. As the teaching model of the education system, modern informatization mainly uses informationized teaching resources and higher English international teaching.

### 3.2. Organizational Structure Measurement Indicators for College English Classroom Teaching Evaluation in an Information Learning Environment

The higher English teaching evaluation index is used as a teaching model for English teachers and students individually, and the input energy from teaching is rationally allocated as an international teaching system. A certain teaching model can be constructed to ensure smooth energy flow and high efficiency. The teacher evaluation system can run the sequence in a healthy manner [14, 15]. In the modern information environment, the teacher evaluation system includes the interaction between the teachers, students, and teaching resources, and detailed teacher learning and classroom learning can explore the learning motivation of students and ensure that the input system energy meets the characteristics of all aspects in these mutual exchanges. The measurement is suitable for the organizational structure of higher English internationalization evaluation to construct teaching evaluation indicators. Teachers and students need to meet the needs of each other, and their mutual adaptability is very high. According to their own teaching activities to supervise each other's work, the way of energy transfer between each other has become more fluent, and the number of energy conversions has increased. On the whole, fitness satisfies the three aspects, namely, purpose fitness, content fitness, and method adaptation. Teaching attitude plays an important role in the evaluation system of higher English teachers. The purpose of different activities, teaching content, and learning attitudes are in line with the teaching levels of both parties.

### 3.3. Resilience Index of College English Classroom Teaching Evaluation in an Information Learning Environment

The resilience of the English curriculum evaluation system refers to the ability of the teaching evaluation system to be threatened by the outside world and to maintain the system's ability to create and function normally. In order to maintain the normal operation of teaching evaluation, the evaluation system can play an overall adjustment role and strengthen the protection elements to reduce the risk. This requires higher English teachers to have a sense of self-reflection in the teaching process and be able to consciously correct the existing risk factors in time. The main influencing factors in the evaluation system are the teaching fatigue of the English teachers in the teaching process, the lack of motivation of students, and the information incompatibility existing in the environment of globalization, and the teaching organization structure is threatened from the outside. This will be caused by teachers' fatigue, the interaction between student's learning and teacher's teaching activities, goals, teaching content, teaching attitudes, and teaching methods that cannot meet their needs. It is not suitable to be applied to the modern information teaching environment. It needs to constantly overcome the existing problems. Teachers and students need to have the ability to reflect, detect the existing dangerous factors, and take corresponding measures to overcome the existing difficulties. This will enable teachers' and students' educational abilities to be effectively used, and the existing risk factors can be detected. The good state of learning motivation and organizational teaching structure is equivalent to the key protective factors in the English classroom evaluation system, in order to effectively promote English teachers, and the embodiment of the education level of the students ensures that the students have better learning ability.

## 4. Realization of Optimization of Higher English Internationalization Education Model and Evaluation System

Constructing a binding parameter index analysis system for higher English internationalization education model and evaluation analysis, using multisource information fusion for higher English internationalization education model and evaluation based on the analysis of big data information system, in order to improve the quantitative assessment ability of higher English classroom scheduling level, we propose a higher English classroom teaching analysis method based on a fuzzy greed algorithm and information fusion, analyze higher English classroom teaching, and transform the evaluation problem into a least-square estimation problem of the *K*-means cluster objective function. The least-squares problem is to find the consistent estimation value of the higher English internationalization education model and the evaluation resource constraint vector *β* so that ‖*Y* − *Xβ*‖ can be minimized, where ‖·‖ is the F-norm in the European algebra norm, and obtains the constraint characteristics of the ability of advanced English classroom scheduling. The entropy feature extraction value of the information is

(6) $$\begin{array}{c} P_{\text{loss}}=1-\frac{1-p_{0}}{\rho }=\frac{p_{0}+\rho -1}{\rho }=\sum_{n=1}^{N}p_{k,n}. \end{array}$$

Given that *d*_*i*_ is the perturbation feature vector for teaching analysis and evaluation, the estimating formula of higher English classroom arranging ability is transformed into the least square solution

(7) $$\begin{array}{c} z\left(t\right)=x\left(t\right)+iy\left(t\right)=a\left(t\right)e^{i\theta \left(t\right)}+n\left(t\right), \end{array}$$

where *x*(*t*) is the real part of the time series for evaluating the distribution of big data, and *y*(*t*) is the imaginary part of the higher English international education model and evaluation constraint index sequence.

Using surrogate data method to randomize the teaching ability of higher English classrooms can also disturb the empirical distribution data of the k^th^ education analysis and evaluation of functional, and obtain the *k*^th^ subgroup, which represents the utilization rate of the resource distribution of higher English classrooms.

(8) $$\begin{array}{c} U_{\text{util}}=\gamma \bar{X}. \end{array}$$

Constructing a hierarchical tree, using big data analysis methods, establishing the main component characteristics of the analysis and evaluation outside the teaching time of higher English classrooms, and using ambiguous close filling methods can solve the similarity of the distribution of educational resources.

(9) $$\begin{array}{c} {\text{Sim}}_{1}\left(d_{i},d_{1j}\right)=\frac{\sum_{k=1}^{M}W_{ik}\times W_{1jk}}{\sqrt{\sum_{k=1}^{M}W_{ik}^{2}}\cdot \sqrt{\sum_{k=1}^{M}W_{1jk}^{2}}}, \end{array}$$

where *d*_*i*_ is the prior distribution feature vector of higher English internationalization education model and evaluation and *d*_1*j*_ is the *K*-means clustering center vector of the first-level big data.

Combining the fusion method of linear correlation characteristics, the clustering, and integration of the index parameters of the higher English classroom teaching evaluation are realized, and the fusion formula of the output education resource information is as follows:

(10) $$\begin{array}{c} P\left(w|x\right)=\frac{P\left(x|w\right)}{P\left(x\right)}. \end{array}$$

If the quantitative recursive feature (*N*(*i*)mod*L*) < *m*, the probability density feature *p*(*i*)=⌊*N*(*i*)/*L*⌋ of the distribution of teaching resources, the higher English internationalization education model, and the evaluation big data stream *X*(*i*) are divided into *p*(*i*) submatrices *N*_*ij*_ × *m* with the size of *X*_*ij*_, and they are aggregated by index parameters, classes, and integration, and compile appropriate teaching evaluation contents, so as to realize the evaluation of international higher English education model.

## 5. Improvement Strategies for Higher English Internationalization Education under the Background of Multi-Source Information Fusion

### 5.1. Adjust Teaching Goals

If information processing methods and big data analysis methods are used to adjust teaching evaluation and resource utilization, the quantitative control of teaching progress will be improved and it will play an important role in the level of planning ability. Therefore, it aims at the background analysis of higher English teaching ability assessment. Because of the influence of many factors, the evaluation of higher English teaching ability first conducts experiments and researches on higher English teaching level, establishes a data system and resource analysis system for higher English teaching level, and uses information combination and clustering solutions to solve higher English. The evaluation of teaching ability and the establishment of the target and statistical system of English teaching ability evaluation can significantly improve the quantitative budget ability of higher English teaching ability evaluation. In the higher English international education model and evaluation index system, the effect of the international education model and evaluation index system is affected by the order of courses. It can be seen from the effect of the order of courses that the arrangement of higher English classrooms in a college is reasonable, and what is the effect of college education. The ranking of higher English classrooms represents the feasibility of the entire class schedule of this college.

### 5.2. Strengthen the Design of Higher English International Education Courses

For the traditional international education model and evaluation index system ability evaluation calculation, there is a situation of inaccurate classification. Based on this situation, research scholars have proposed an international education model and evaluation index system ability evaluation calculation method on the combination of fuzzy greedy calculation method and information. First, set up a research system for constrained parameter indicators, then use quantitative recursive methods to evaluate the ability of the data information system to achieve the ability to control the acquisition of characteristic resources, complete the classification and summary of the index parameters of the international education model and the ability of the evaluation index system, and edit the corresponding the teaching resource plan. Complete the evaluation of the ability of the evaluation index department. Using this calculation method to carry out the evaluation of the ability of the international education model and the evaluation index system, the information integration and analysis ability is high, the accuracy of the teaching ability evaluation is greatly improved, and the efficiency of the use of educational resources is improved.

### 5.3. Improve the Teaching Test and Evaluation System

For a long time, the evaluation of China's higher English internationalization education is based on final evaluation, with final exams and CET-4 and CET-6 as the main test methods, but students' evaluation of the English learning process is relatively neglected. Do not pay attention to the assessment and evaluation of students' learning methods, knowledge application ability training, and other key skills. CET-4, CET-6, CET-4, and CET-8 all emphasize achievement and pass rate. It has brought many negative effects to students' English learning. The question type of the college English test has a big flaw in its design. Not only is there a big deviation in the basic internationalization of college English education, but also the review of many contents cannot fully reflect the comprehensive language application ability of college students. In particular, the review of oral skills and translation skills has weakened. The phenomenon of dumb English with poor ears is still relatively serious. Therefore, it is necessary to reform the current higher English international education testing and evaluation system. On one hand, increase the proportion of formative evaluation and ask students to speak, read, write, and perform comprehensive test translation and other language skills to promote students' application skills of English knowledge. On the other hand, make corresponding changes in the form of English examination questions and improve the effectiveness and accuracy of the review process. If objective problems can be reduced, questions such as conversational tests and subjective questions will be added, focusing on cultivating students' ability to use English language thinking skills and English knowledge to solve practical problems.

### 5.4. Pay Attention to the Construction of the Teaching Staff

In order to further accelerate the internationalization of higher English education and the process of internationalization of education, we must pay attention to the direct impact of the construction of the teaching staff. In the context of multisource information integration in higher education, the construction of the teaching team is ensured. The key to the smooth progress of the reform of higher English international education is to improve the professional quality of high school English teachers and to further improve the education level and quality of education. In order to better meet our country's actual needs for training international English talents. At present, college English teachers regularly participate in educational seminars, and training is the main way to build the teacher team. However, this is obviously insufficient for cultivating new international talents. On the basis of strengthening in-service teacher training, the university encourages students to participate in foreign language education seminars at home and abroad. If conditions permit, teachers can be given more opportunities for overseas exchanges and training. Expand the horizons of teachers' international education and form the ability of international thinking and practice in English education. In addition, on the basis of accumulating their own professional knowledge, college English teachers have been extensively involved in pedagogy, linguistics, psychology, sociology, anthropology, and other related subject knowledge, improving personal comprehensive quality and accelerating the accumulation and integration of and subject experience, so as to improve the quality of English international education.

## 6. Experimental Process and Results

This experiment will use this indicator system to analyze the results of the experiment. First, establish a hierarchy, based on the levels and elements of the learning (*a*1) part of the higher English international education model in Table 1; English learning input (*b*1) and English learning output (*b*2) are contained in it, and *c*1 is the visible learning level indicator. Adopt the sum of compulsory and elective hours, and the evaluation criteria are over 150A, 120–150B, 90–120C, 60–90D, E under 60, converted into a percentage system A 100 points, B 85 points, C 70 points, D 55 points, and E 40 points; *c*2, the invisible learning indicator calculates the level and number of students participating in competitions, participation in English-related lectures and activities, participation in international academic exchanges, and English-related practical activities, which are converted into a hundred-point system; *c*3 indicators are degree courses and evaluation standards. It is a percentile system with a score of 7 : 3 on the roll and usual; *c*4 is the accumulation of other output such as awards in the National College English Contest and submission and publication of English papers (assigned according to ISTP, EI equal levels), etc. and is converted into a percentile system. Secondly, the corresponding questionnaire was compiled, and opinions were solicited from 20 teachers engaged in English teaching for non-English major graduate students to confirm the final judgment matrix and form the weight coefficient, as shown in Figures 2–4 and Tables 1–3.

When *λ*max = 1.5, when CI = 0 is satisfied, the obtained matrix has complete consistency (Figure 2).

When *λ*_max_ = 2.0, when CI = 0 is satisfied, the obtained matrix is completely consistent (Figure 3).

When *λ*_max_ = 2.5, when CI = 0 is satisfied, the obtained matrix has complete consistency (Figure 4).

The results of the 2019 higher English internationalization teaching courses are selected in order of 67–74 points, of which there are 50 students, 25 boys and 25 girls. The selected student targets have no significant difference in age. The detailed distribution is shown in Figure 5. As shown, in the evaluation of the quality of the teaching model, this single result obviously cannot be used to objectively evaluate the 50 students with insignificant differences in scores.

From the analysis of the experimental results, it can be seen that the higher English internationalization education index assessment constructed in this article has a good degree of discrimination, can more reasonably evaluate the higher English internationalization teaching ability, and can also make the evaluation process more objective and scientific. This provides a scientific basis for follow-up teaching quality evaluation.

## 7. Conclusions

According to the above analysis, it can be seen that there are many problems in the teaching process of higher English international education based on the multisource information fusion algorithm. The English teachers of colleges and universities need to reform according to the teaching level, mainly from the English teaching goals and English courses. Design standards, teaching content compilation, teaching quality evaluation, and English teacher team construction are analyzed from different perspectives to realize the adjustment and innovation of previous higher English nationalization teaching programs and effectively enrich the role and functions of higher English international education. Improve the teaching level of English internationalization and better adapt to the development trend of the internationalization of higher education and economic globalization.

## Figures and Tables

**Figure 1:** Multisource information fusion diagram of college English in higher vocational colleges.

**Figure 2:** *a*-*b* matrix diagram.

**Figure 3:** *b*_1_-*c* matrix diagram.

**Figure 4:** *b*_2_-*c* matrix diagram.

**Figure 5:** Distribution of English comprehensive ability assessment results.

**Table 1:** *a*-*b* comparison judgment matrix.

*a*_1_	*b*_1_	*b*_2_	*w*
*b*_1_	1.5	1.5	1
*b*_2_	1.5	1.5	1

**Table 2:** *b*_1_-*c* comparison judgment matrix.

*b*_2_	*c*_1_	*c*_2_	*w*
*c*_1_	1.5	1.5	1
*c*_2_	0.5	1.5	1

**Table 3:** *b*_2_-*c* comparison judgment matrix.

*b*_2_	*c*_3_	*c*_4_	*w*
*c*_3_	1.5	4.5	1.3
*c*_4_	0.5	1.5	0.7

## Data Availability

Data sharing does not apply to this article as no datasets were generated or analyzed during the current study.
